# Comparative Efficacy of Chinese Patent Medicines for Clearing Heat and Dampness in the Treatment of NAFLD: A Network Meta-Analysis of Real-World Evidence

**DOI:** 10.1155/2022/4138555

**Published:** 2022-07-31

**Authors:** Yuan Xu, Yan Wang, Xiao-jun Gou, Man Wang

**Affiliations:** ^1^School of Pharmacy, Shaanxi University of Traditional Chinese Medicine, Xianyang 712046, Shaanxi, China; ^2^Central Laboratory, Baoshan District Hospital of Integrated Traditional Chinese and Western Medicine of Shanghai, Shanghai University of Traditional Chinese Medicine, Shanghai 201999, China; ^3^Pharmacy Department, Shanghai Putuo District Liqun Hospital, Shanghai 200333, China; ^4^Nutriology Department, Shanghai Fengxian District Central Hospital, Shanghai 201499, China

## Abstract

**Background:**

Nonalcoholic fatty liver disease (NAFLD) has emerged as the most common chronic liver disease, as well as a worldwide medical problem with a substantial socioeconomic burden. In China, Chinese patent medicines (CPMs) have been widely utilized as promising and effective therapy options for NAFLD. Traditional Chinese medicine (TCM) is a particular kind of medical science reliant on real-world clinical practices and evidence. Therefore, using the real-world data extracted from pragmatic randomized controlled trials (PRCTs) have more reference value for the application of CPMs in NAFLD.

**Method:**

Six databases were searched from their inception up to March 18, 2022. The methodological quality of the included study was evaluated by the Cochrane risk-of-bias tool. Then, The STATA 13.0 program was then used to do a network meta-analysis (NMA) of real-world studies. The surface under the cumulative ranking curve (SUCRA) probability values were applied to rank the examined treatments.

**Results:**

Forty-three PRCTs (4997 cases in total) were identified. Da-Huang-Li-Dan capsule (DHLD), Dan-Ning tablet (DN), Dang-Fei-Li-Gan-Ning capsule (DFLGN), Qiang-Gan capsule (QG), and Hua-Zhi-Rou-Gan granule (HZRG) were among the five CPMs tested. As far as the clinical effective rate of the primary outcome index was concerned, the top three CPMs were DN + CDs: OR = 0.19, 95% CIs: 0.12, 0.31 (SUCRA: 81.8%); DFLGN + CDs: OR = 0.21, 95% CIs: 0.09, 0.46 (SUCRA: 74.9%), and DHLD + CDs: OR = 0.26, 95% CIs: 0.10, 0.67 (SUCRA: 61.1%). In terms of liver function index, DN + CDs ranked first in ALT index: MD = 15.81, 95% CIs: 10.05, 21.57 (SUCRA: 85.5%), DFLGN + CDs ranked first in AST index: MD = 14.94, 95% CIs: 4.77, 25.11 (SUCRA: 83.6%), HZRG + CDs ranked first in TC index: MD = 0.53, 95% CIs: 0.28, 1.03 (SUCRA: 87.1%) and TG index: MD = 1.8, 95% CIs: 1.41, 2.30 (SUCRA: 79.9%).

**Conclusion:**

Using CPMs as a coadjuvant treatment might be positive efficacious intervention from which patients with NAFLD will derive benefits. When it came to the clinical effective rate and other outcomes, DN + CDs demonstrated a significant improvement in individuals with NAFLD.

## 1. Introduction

Nonalcoholic fatty liver disease (NAFLD) has become the most prevalent liver metabolic disease, affecting approximately 1.7 billion individuals around the world [1–3]. NAFLD can be classified as simple steatosis and nonalcoholic steatohepatitis (NASH), cirrhosis, and hepatocellular carcinoma based on its pathological stages [4, 5]. In the United States, these increased trends in the prevalence and incidence of NAFLD may also be seen in children and adolescents. Similar increases have been observed in Europe, China, India, and other regions of the world. As a result, NAFLD has grown into a worldwide medical problem with severe socioeconomic implications [6].

Chinese patent medicines (CPMs) have been found in studies to have a greater therapeutic impact, less toxic and side effects, and high safety when used in combination with CDs. CPMs have been widely used as adjuvant therapy for NAFLD in China in recent years [7–9]. We discovered that five CPMs, including Da-Huang-Li-Dan capsule (DHLD), Dan-Ning tablet (DN), Dang-Fei-Li-Gan-Ning capsule (DFLGN), Qiang-Gan capsule (QG), and Hua-Zhi-Rou-Gan granule (HZRG), have been widely used in NAFLD of the dampness and heat accumulation type due to their outstanding effects, based on clinical medication experience and previous searches in electronic databases. Systematic reviews have demonstrated their effectiveness [7, 10, 11]. Traditional Chinese medicine (TCM) has no term for “fatty liver,” although it can be characterized as “hypochondriac pain,” “accumulation,” or “jaundice” based on clinical symptoms. Fatty liver is caused by overeating fat and spicy foods, endogenous damp evil, long-term stagnation or abnormal transportation and transformation of spleen and stomach functions, endogenous dampness, and turbidity. Therefore, clearing heat and dampness is an important treatment in the treatment of NAFLD.

When CPMs are used in conjunction with traditional CDs, clinical symptoms can be considerably improved. However, it is impossible to accurately and thoroughly examine the advantages and drawbacks of numerous therapies using pairwise meta-analysis. The network meta-analysis (NMA) is a new sort of evidence-based medical statistical approach which allows for simultaneous examination of the efficacy of many interventions by comparing direct and indirect evidence and ranking the efficacy of various therapies to make a conclusion [12, 13]. Another important characteristic of NMA is that it may rate each CPM based on its efficacy, assisting physicians in making the optimal treatment options. In recent years, the concept of real-world research has emerged, and real-world data and evidence have become more and more important in the field of medical and health decision-making. Randomized controlled trial is recognized as the “gold standard” for evaluating the effectiveness of intervention measures, which can be divided into exploratory randomized controlled trials and pragmatic randomized controlled trials (PRCTs). TCM is an empirical medicine that mainly relies on case reports and clinical experience summaries. Through the evidence in the real world, it can promote the personalized application of TCM diagnosis and treatment rules, so the reference significance based on PRCTs for TCM is more important. Therefore, the purpose of this study is to evaluate the clinical efficacy of various CPMs combined with CDs by combining big data with real-world data and provide further evidence for rational drug selection.

## 2. Materials and Methods

This study was registered on the PROSPERO (International Prospective Register of Systematic Reviews) and the registration ID is CRD42022323979. The present report follows the Preferred Reporting Items for Systematic Review and Meta-analysis (PRISMA) Protocols guidelines [14].

### 2.1. Data Sources and Search Strategy

From the establishment of each electronic database to March 18, 2022, PRCTs using methods of clearing heat and removing dampness to treat NAFLD were searched in the following 6 electronic databases: PubMed, Embase, Cochrane Library, the Chinese National Knowledge Infrastructure, Wanfang Database, and Weipu Database. No restriction on the publication year, language, or blinding methods were implemented.

Searching for the following terms: (“Complementary Therapies” OR “Complementary and alternative therapies” OR “Alternative Medicine” OR “Alternative Therapies” OR “Complementary Medicine” OR “Herbal therapy” OR “Therapy, Alternative” OR “Therapy, Complementary” OR “Therapies, Alternative”) AND (“Non-alcoholic Fatty Liver Disease” OR “Steatohepatitis, Nonalcoholic” OR “Nonalcoholic Steatohepatitides” OR “NAFLD”) AND (“clinical trial” OR “randomized controlled trial” OR “randomized controlled trial”). In our literature search, we did not define the language or status of the papers. Additional references were found by manually searching bibliographies of included trials and associated reviews.

### 2.2. Criteria for Literature Inclusion

Clinical studies using CPMs for clearing heat and dampness in the treatment of NAFLD were included in this network meta-analysis. Trials were excluded if

1. there was no control group or there was a combination with other drugs;
2. trials on effective analysis data could not be obtained;
3. they were reviews, observational studies, cross-sectional, case reports, conference papers, meta-analyses, experience sharing, animal trials, etc.

Studies that matched the following criteria were considered eligible:

1. PRCTs that evaluated the efficacy of CPMs combined with CDs were included.
2. All of the patients were diagnosed with NAFLD using the Guidelines of prevention and therapy for NAFLD [15].

### 2.3. Outcomes

Clinical effectiveness was defined as the primary outcome. The improvement in clinical symptoms of patients before and after treatment was used to assess the clinical effect of medications, which might better reflect the therapeutic effect of pharmaceuticals. According to the degree of alleviation, symptoms were classed as effective or ineffective. Other outcomes included liver function: the Alanine aminotransferase (ALT) and aspartate aminotransferase (AST), and also blood lipid indexes such as triglyceride (TG) and total cholesterol (TC).

### 2.4. Study Selection and Data Extraction

Data extraction was performed independently by two reviewers who participated in training and calibration exercises using Endnote X9 to do the screening. If there was a disagreement, they worked it out via conversation or had it evaluated by a third party. The third party also employed a standardized screening form and did calibration exercises prior to the screening procedure.

The researchers gathered information on the following features for all qualifying trials:

1. Basic information (first author, title of study).
2. Participant characteristics (sample size, gender, and age).
3. Measures of prevention and control (dosage form, dose, and duration).
4. Risks of bias investigation.
5. Outcome Measures

### 2.5. Assessment of Literature Quality

Two reviewers independently assessed the risk of bias for PRCTs using the Cochrane Collaboration's “risk of bias” technique. The Cochrane handbook was used to develop the assessment criteria [16]. The two reviewers' disagreement was resolved through discussion. If there is a disagreement between two reviewers, the paper will be sent to a third person for review.

### 2.6. Statistical Analysis

The Cochrane Collaboration's RevMan 5.3 software was used to conduct statistical analyses of literature quality. Calculations and graphs were generated using STATA 13.0 software, the Bayesian random-effects NMA using Markov-chain Monte Carlo simulation. After an initial burn-in of 20,000 iterations and a thinning interval of 10, the random-effects model for outcomes was chosen in the NMA, which was run with four chains and 50,000 simulated iterations. We calculated mean differences (MD) with corresponding 95% credible intervals (CIs) for continuous outcomes and odds ratios (OR) with corresponding 95% CIs for dichotomous. We divided multiarm studies into two-arm trials, if there were any. The Chi-squared test was used to determine the degree of heterogeneity between studies [17]. If the inconsistency was not significant in direct and indirect comparisons, the consistency model was used for further analyses. The premise of consistency between direct and indirect evidence was not used in this NMA due to nonclosed loops.

## 3. Results

### 3.1. Selection and Identification of Studies

A total of 6119 possibly relevant trials were retrieved, with 1223 trials remaining after 4896 duplicates and irrelevant trials were removed. Following a review of the titles and abstracts, 1014 publications were eliminated because they did not fulfill the inclusion criteria, and 209 trials were found to meet the planned standards for further evaluation after reading the complete text. Finally, 43 studies [18–60] were included in the meta-analysis.  Figure 1 depicts the PRISMA flow diagram of the literature retrieval process. All of the trials that were included in the study were published as complete publications.

### 3.2. Included Study Characteristics

Table 1 summarized the basic characteristics of the 43 trials, and a total of 4997 patients were included. In these 43 trials. 3 trials used DHLD + CDs vs. CDs [18–20], 16 trials used DN + CDs vs. CDs [21–36], 4 used DFLGN + CDs vs. CDs [37–40], 8 used QG + CDs vs. CDs [41–48], and 12 used HZRG + CDs vs. CDs [49–60]. Among these PRCTs, control groups have been treated with CDs like statin lipid-lowering agents, anti-inflammatory, hypoglycemic drugs, and nutritional support. The statin lipid-lowering agents mainly include atorvastatin, simvastatin, and rosuvastatin as a single treatment or a combination of treatments. The experimental group's intervention was one of the CPMs included in the control group's intervention. The therapy lasted from around 6 to 24 weeks. Table 1 shows the study's features in detail, and Figure 2 shows the comparative links between each intervention and each result.

### 3.3. Methodological Quality Assessment

Among the 43 PRCTs, 8 studies used the random number method or computer to create random number words, with low-risk bias, 16 studies used outpatient order or a period of hospitalization, so there was high-risk bias, and 4 studies used the method of distribution of low-risk bias. Because none of the 43 PRCTs indicated subject and researcher blinding or evaluator blinding to the result, they were all rated as “unclear”. 4 of the studies did not explain the reasons for the missing data, the remaining 27 studies had no missing data, and 12 studies were unclear. We were unable to gather thorough information on the remaining two aspects, selective reporting outcomes, and other biases. Therefore, we rated them all as “unclear.” Figures 3 and 4 provide the exact findings of the bias risk assessment for all PRCTs.

### 3.4. Results of the NMA

#### 3.4.1. Clinical Effect

Clinical effect was reported in 43 trials, in which 3 used DHLD + CDs vs. CDs [18–20], 16 used DN + CDs vs. CDs [21–36], 4 used DFLGN + CDs vs. CDs [37–40], 8 used QG + CDs vs. CDs [41–48], and 12 used HZRG + CDs vs. CDs [49–60].

There were 43 comparisons in the network of comparisons in Table 2, and DHLD, DN, DFLGN, QG, HZRG combined with CDs improved the clinical effective rate more significantly than CDs alone (DHLD + CDs : OR = 0.26, 95% CIs: 0.10, 0.67; DN + CDs : OR = 0.19, 95% CIs: 0.12, 0.31; DFLGN + CDs : OR = 0.21, 95% CIs: 0.09, 0.46; QG + CDs : OR = 0.44, 95% CIs: 0.27, 0.74; HZRG + CDs : OR = 0.27, 95% CIs: 0.17, 0.43). Notably, there were significant differences between DN + CDs and QG + CDs.

The SUCRA values in Table 3 and Figure 5 indicated that DN + CDs was the best therapy, DFLGN + CDs was second, and DHLD + CDs was third.

#### 3.4.2. The Level of ALT

40 PRCTs (3 used DHLD + CDs vs. CDs [18–20], 15 used DN + CDs vs. CDs [21–29, 31, 32, 34, 35], 4 used DFLGN + CDs vs. CDs [37–40] 7 used QG + CDs vs. CDs [41–48], and 11 used HZRG + CDs vs. CDs [49–59]) with five treatments reported the TG. The results of the pairwise meta-analysis are shown in Table 4. According to Table 4, DN, QG, HZRG combined with CDs (DN + CDs : MD = 15.81, 95% CIs: 10.05, 21.57; QG + CDs : MD = 12.20, 95% CIs: 4.42, 19.99; HZRG + CDs : MD = 11.23, 95% CIs: 4.85, 17.62) were more effective than CDs alone; there were no significant differences between each comparison of different CPMs.

The SUCRA values in Table 3 and Figure 5 indicated that DN + CDs was the optimal treatment, QG + CDs was the second, and HZRG + CDs was the third.

#### 3.4.3. The Level of AST

35 PRCTs (3 used DHLD + CDs vs. CDs [18–20], 11 used DN + CDs vs. CDs [21, 23–25, 27, 29–33, 35], 3 used DFLGN + CDs vs. CDs [37–40] 7 used QG + CDs vs. CDs [41, 43–48], and 11 used HZRG + CDs vs. CDs [49–59]) with five treatments reported the AST. The results of the pairwise meta-analysis are shown in Table 5. According to Table 5, DHLD, DN, DFLGN, HZRG combined with CDs (DHLD + CDs : MD = 13.45, 95% CIs: 3.61, 23.28; DN + CDs : MD = 7.43, 95% CIs: 1.95, 12.91; DFLGN + CDs : MD = 14.94, 95% CIs: 4.77, 25.11; HZRG + CDs : MD = 11.63, 95% CIs: 6.25, 17.02) were more effective than CDs alone; QG + CDs did not perform more remarkable than CDs alone.

The SUCRA values in Table 3 and Figure 5 indicated that DFLGN + CDs was the optimal treatment, DHLD + CDs was the second, and HZRG + CDs was the third.

#### 3.4.4. The Level of TC

TC was estimated in 37 PRCTs, in which 3 used DHLD + CDs vs. CDs [18–20], 14 used DN + CDs vs. CDs [21–32, 34, 35], 4 used DFLGN + CDs vs. CDs [37–40], 5 used QG + CDs vs. CDs [41, 43, 44, 47, 48], and 11 used HZRG + CDs vs. CDs [49–59]. The results of the pairwise meta-analysis are shown in Table 6. According to Table 6, DN, DFLGN, QG, HZRG combined with CDs (DFLGN + CDs : MD = 0.84, 95% CIs: 0.38, 1.83; QG + CDs : MD = 1.41, 95% CIs: 0.65, 3.08; HZRG + CDs : MD = 0.53, 95% CIs: 0.28, 1.03) had better treatment than CDs alone, and there were no significant differences among other groups.

The SUCRA values in Table 3 and Figure 5 indicated that HZRG + CDs was the optimal treatment, DFLGN + CDs was the second, and DHLD + CDs was the third.

#### 3.4.5. The Level of TG

37 PRCTs (3 used DHLD + CDs vs. CDs [18–20], 13 used DN + CDs vs. CDs [21–29, 31, 32, 34, 35], 4 used DFLGN + CDs vs. CDs [37–40] 6 used QG + CDs vs. CDs [41–44, 47, 48] and 11 used HZRG + CDs vs. CDs [49–59]) with five treatments reported the TG. The heterogeneity results of the pairwise meta-analysis are shown in Table 7. According to Table 7, DHLD, DN, DFLGN, QG, HZRG combined with CDs (DHLD + CDs : MD = 1.52, 95% CIs: 1.04, 2.22; DN + CDs : MD = 1.63, 95% CIs: 1.34, 1.98; DFLGN + CDs : MD = 1.44, 95% CIs: 1.03, 2.01; QG + CDs : MD = 1.69, 95% CIs: 1.30, 2.21; and HZRG + CDs : MD = 1.8, 95% CIs: 1.41, 2.30) were more effective than CDs alone, and there were no significant differences among other groups.

In Table 3 and Figure 5, the SUCRA values suggested that HZRG + CDs was the optimal treatment, QG + CDs was the second, and DN + CDs was the third.

### 3.5. Funnel Plot Characteristics

Figure 6 shows comparison adjusted funnel plots for various outcomes. Results TG was the only funnel plot without bias. The majority of the dispersion points were positioned in the middle and top half of the inverted triangle. As a result, there was no bias due to publishing. The funnel plot was asymmetric, indicating a limited sample size and publication bias, among other outcomes.

## 4. Discussion

A total of 43 PRCTs involving 4997 individuals were included in the study. DHLD, DN, DFLGN, QG, and HZRG are five CPMs that have been found in the therapy of NAFLD. Because of the heterogeneity, the Mantel-Haenszel random-effects model was utilized for the meta-analysis. Due to the nonclosed loops in this NMA, the assumption of consistency between direct and indirect evidence was not used. This network meta-analysis found five interesting outcomes: clinical effective rate, ALT, AST, TC, and TG. In terms of clinical effective rate, the results showed that DHLD, DN, DFLGN, QG, and HZRG coupled with CDs had a better impact than CDs alone. We may infer that DN + CDs was the best in terms of clinical response rate and improvement based on SUCRA values. We can conclude that DN + CDs was the best in terms of clinical response rate and ALT improvement, DFLGN + CDs was the best in terms of AST improvement, and second in terms of clinical response rate and TC improvement, and HZRG + CDs was the best in terms of TC and TG outcomes improvement. However, it rated worse in other outcome indicators. As a consequence of the above analyses, we conclude that DN + CDs might be a potential therapy option. However, as can be observed from the funnel plot, the outcome indicator had a modest degree of bias in addition to TG, and other outcome indicators had a large degree of bias due to the existence of low-quality PRCTs. Thus the evidence strength of other outcomes may be reduced.

The pathogenesis of NAFLD cannot be clearly explained. The hypothesis widely accepted by scholars is the pathogenesis of “second hit;” the “first hit” induces fat accumulation in hepatocytes and increases hepatic uptake of free fatty acids. There are still many controversies about the “second hit.” Jung et al. [61] believed that liver cell damage caused by oxidative stress and inflammation is a key factor in the pathological process from simple fat accumulation to severe liver disease. Another mechanism that leads to the pathogenesis of NAFLD emerging factor is the gut microbiota imbalance. Le et al. [62], with the same germ-free mice fed a high-fat diet, by inoculating fecal bacteria to isolate pathological and normal mice, found that in mice vaccinated with pathological bacterial isolates in adipose sex hepatitis, the normal mice fat only showed the low degree of degeneration. The reason for this phenomenon may be that the gut microbiota increased circulating bacterial endotoxins and triggers a cascade of proinflammatory cytokines in the liver. It is also possible that the gut microbiota leads to abnormal metabolism of endogenous metabolites, which increases fat production in the liver and leads to NAFLD. As clinical and basic research continues to deepen, the mechanisms of NAFLD are still being defined. NAFLD is an extremely complex and subtle disease, representing the convergence of various pathways, risk factors, and external influences, which are not uniform in all patients [63]. The only two treatment options currently available for the treatment of NAFLD are control of risk factors (diabetes, hypertension, and dyslipidemia) and weight loss [64]. Control energy intake of the surplus is a more effective way to lose weight. Excessive fat accumulation has resulted in a net in the form of triglycerides in the liver, too much energy over white fat storage limit at the same time, the excess energy accumulated in the liver and eventually promotes the emergence and development of NAFLD. Although excessive use of any food can lead to the occurrence of NAFLD, excessive intake of monosaccharides and disaccharides can activate the heparin regeneration process and further aggravate NAFLD metabolized as triglyceride [6].

Because there is no authorized medication specifically for NAFLD, the primary treatment for the disease is now lifestyle modification [65]. However, most individuals find it difficult to maintain a healthy lifestyle, whether it be via physical exercise or food limitations. As a result, researchers are working to develop novel treatments for NAFLD. So far, a variety of medications have been explored for the treatment of NAFLD. Although the following therapeutic classes may have demonstrated advantages in treating NAFLD, we are aware that finding a pharmacological treatment that targets a wide range of the previously reported complicated physiopathology of NAFLD is challenging. As a result of the multicomponent, multitarget, and multipathway nature of TCM, it has a lot of promise in treating NAFLD and avoiding disease development. Damp-heat accumulation syndrome is one of the main types of NAFLD. Because the etiology of NAFLD is not controlled by diet or exogenous damp-heat epidemic toxin, which leads to endogenous damp evil and phlegm turbidity, it is often used to treat NAFLD by clearing heat and dampness.

There is now a large body of data that CPMs can effectively improve NAFLD. Four weeks of QG therapy in rats with NAFLD caused by a high-fat diet reversed leptin resistance and reduced lipid accumulation and inflammation in the liver [66]. There was also evidence that CPMs were helpful in avoiding NASH, with the underlying probable processes being linked to the interplay of gut microbiota and BA metabolism, as well as TGR5-mediated NF-*κ*B suppression [67].

DN as a TCM formula has been broadly applied in treating hepatobiliary diseases, especially gallbladder stones, cholecystitis, and fatty liver syndromes in clinical trials [68, 69]. DN including Dahuang (*Rhei radix* et Rhizoma), *Hu zhang* (*Polygoni cuspidati* Rhizoma et Radix), Chenpi (Citri Reticulatae Pericarpium), Qingpi (Vatica mangachapoi Blauco), Baimaogen (*Rhizoma imperatae*), Yujin (Radix *Curcumae aromaticae*), Jianghuang (*Curcumae radix*), and Shanzha (*Crataegi fructus*). It has the function of clearing heat and soothing the liver and promoting gallbladder. Dahuang is the monarch medicine of DN, which has the effect of purging heat and clearing intestines, cooling blood, detoxification, and removing blood stasis; Huzhang clears away heat and toxic materials, Baimaogen clears heat and cools blood, both of which are ministerial medicines; Chenpi and Qingpi are the assistant medicines to reconcile the spleen and stomach; Yujin soothes the liver and promotes gallbladder; Shanzha can eliminate stagnation and blood stasis. One study showed that DN could attenuate the development of NAFLD and associated metabolic diseases in HFD-induced NAFLD mice. DN can inhibit the expression of SREBP-1 and SREBP-2 and their downstream genes might be the possible mechanisms of inhibiting liver fat production and cholesterol synthesis [70].

In this article, NMA is strictly complied with PRISMA guideline. Traditional clinical research, represented by RCT, investigates the therapeutic efficacy of intervention measures in an ideal environment of strict control and has high internal authenticity. However, because the subjects of RCT are highly homogeneous and the intervention measures are excessively uniform and standardized, the result is that RCT is divorced from the real clinical practice environment, and the extrapolation of research conclusions to clinical practice may face challenges. However, the medical practice of TCM treats patients as a whole, which is the earliest system of individualized medical treatment. It is difficult to analyze TCM's therapeutic effect using a single study design type due to its uniqueness and complexity, which necessitates the flexibility to reflect objective reality while maintaining scientific rigor when evaluating the curative effect of TCM. Real-world research may properly reflect these qualities and give a novel way and methods for evaluating the clinical effect of TCM and collecting evidence. Our findings may provide evidence for the efficacy of CMPs in the treatment of NAFLD and further, indicate the possibility of obtaining clinical significance from CMPs in NAFLD patients.

Three advantages might help to boost the study's credibility. First, as far as we know, this is the first NMA to compare and rate the effectiveness of several CPMs for the treatment of NAFLD. Second, these findings may help physicians in making better treatment decisions for NAFLD. More critically, the ALT, AST, TC, and TG markers were examined in addition to the clinical effectiveness. The most significant transaminases are ALT and AST. ALT and AST levels in the blood are elevated when the liver is injured. The liver primarily produces TG, TC, and phospholipids, which are secreted and delivered into the bloodstream as very low-density lipoprotein for utilization by other tissues and organs [71]. When the quantity of TG produced by the liver exceeds the liver's ability to produce and release extremely low-density lipoprotein, TG is accumulated in liver cells, resulting in NAFLD [72].

However, there are various limitations to consider when understanding our findings. To begin with, the quality of the PRCTs included in this research is low. All PRCTs were conducted in China, and data from clinical research conducted in other languages was insufficient. None of the 43 papers included use the blind approach, and the majority of publications do not offer enough information, such as the randomization procedure, resulting in selection and reporting bias. Second, TCM dialectical diagnosis is a subjective process that might result in misdiagnosis or other biases. Third, the study lacks a planned follow-up, resulting in an erroneous assessment of critical outcome markers such as long-term therapeutic effectiveness. Furthermore, a substantial sample directly comparing the two CPMs was lacking. The fact that various CPMs have varying sample sizes reduces the strength of the evidence supporting the outcomes. A subgroup study based on background disorders, distinct forms of NAFLD, treatment duration, and CDs treatment measures are required. In addition, no subgroup analysis is challenging since the already included studies could not be accurately classified.

Meta-analyses give evidence-based treatment recommendations for clinics. Therefore, well-designed studies are critical. To increase methodological quality, higher-quality and larger-sample PRCTs should be registered in advance. Furthermore, it is recommended that researchers supply as much information on the baseline features as feasible. In the future, more rigorous clinical trials will be necessary to demonstrate the positive effects of CPMs paired with CDs for NAFLD patients.

## 5. Conclusion

In conclusion, the study discovered that CPMs might be effective as a coadjuvant treatment for patients with NAFLD of the dampness and heat accumulation type. In terms of enhancing the clinical effective rate of NAFLD, DN + CDs performed better. In terms of lowering TC and TG levels, HZRG + CDs proved to be more valid. In patients with NAFLD, DN + CDs demonstrated an outstanding improvement in terms of the clinical effective rate and other outcomes. However, owing to the study's limitations, the findings need to be confirmed by further high-quality, large-sample multicenter PRCTs and stronger head-to-head comparative trials. Meanwhile, CPMs safety should be closely monitored and reported.

## Figures and Tables

**Figure 1:** Flow diagram of study inclusion.

**Figure 2:** Network graph of the different outcomes. (a) Clinical effective rate, (b) Alanine aminotransferase (ALT), (c) Aspartate aminotransferase (AST), (d) Serum total cholesterol (TC), (e) Triglyceride (TG).

**Figure 3:** Risk-of-bias graph.

**Figure 4:** Risk-of-bias summary.

**Figure 5:** SUCRA plot for all different outcomes. (a) Clinical effective rate, (b) Alanine aminotransferase (ALT), (c) Aspartate aminotransferase (AST), (d) Serum total cholesterol (TC), (e) Triglyceride (TG).

**Figure 6:** Funnel plot. (a) Clinical effective rate, (b) Alanine aminotransferase (ALT), (c) Aspartate aminotransferase (AST), (d) Serum total cholesterol (TC), (e) Triglyceride (TG).

**Table 1:** Basic characteristics of the included studies.

No.	Literature source	Sample (treatment/control)	Gender			Age (years)		Course (week)	Contrast drugs		Outcome indicators
		*T*	*C*	*M*	*F*	*T*	*C*		*T*	*C*	
1	Li xiangyang (2021)	62	62	71	53	44.44 ± 9.67	44.87 ± 9.58	12	Da-huang-Li-Dancapsule + CDs	CDs	Clinical effective rate, ALT, AST, *γ*-GT, TC, TG
2	Li na (2021)	40	39	47	32	51.91 ± 7.52	51.49 ± 7.04	12	Da-huang-Li-Dancapsule + CDs	CDs	Clinical effective rate, ALT, AST, *γ*-GT, TC, TG, LDL, HDL
3	Wang zhengyan (2020)	43	43	53	33	—		12	Da-huang-Li-Dancapsule + CDs	CDs	Clinical effective rate, ALT, AST, *γ*-GT, TC, TG, LDL, HDL
4	Zhang yu (2018)	35	35	38	32	56.8 ± 6.5		12	Dan-ning tablet + CDs	CDs	Clinical effective rate, ALT, AST, TC, LDL
5	Tao yingjie (2018)	29	29	24	34	45.36 ± 11.54		12	Dan-ning tablet + CDs	CDs	Clinical effective rate, AST, TC, LDL, *γ*-GT
6	Lv junning (2017)	47	46	49	44	26～65	28～66	12	Dan-ning tablet + CDs	CDs	Clinical effective rate, ALT, TC, TG, TBIL
7	Yi ying (2018)	20	20	23	17	45.8 ± 2.9	45.2 ± 2.5	12	Dan-ning tablet + CDs	CDs	Clinical effective rate, ALT, TC, TG, TBIL
8	Xiang fangfei (2019)	39	39	47	31	40.76 ± 2.33	41.63 ± 2.16	12	Dan-ning tablet + CDs	CDs	Clinical effective rate, ALT, AST,
9	Gao ying (2017)	44	44	47	41	43.54 ± 6.43	43.57 ± 6.45	12	Dan-ning tablet + CDs	CDs	Clinical effective rate, ALT, AST, *γ*-GT, TC, TG, LDL, HDL, TBIL
10	Guo zhenying (2018)	66	66	72	60	44.36 ± 8.49	43.74 ± 7.89	12	Dan-ning tablet + CDs	CDs	Clinical effective rate, ALT, AST, *γ*-GT, TC, TG, LDL, HDL, TBIL
11	Peng lirui (2015)	25	25	36	14	51.7 ± 12.3	53.7 ± 13.3	12	Dan-ning tablet + CDs	CDs	Clinical effective rate, ALT, AST, TC, TG
12	Wang yujing (2019)	51	51	55	47	44.0 ± 3.3		12	Dan-ning tablet + CDs	CDs	Clinical effective rate, ALT, AST, TC, TG
13	Li xiaoqing (2019)	32	30	22	40	42.38 ± 10.85	43.37 ± 11.15	12	Dan-ning tablet + CDs	CDs	Clinical effective rate, ALT, AST, *γ*-GT, TC, TG, LDL, HDL, TBIL
14	Feng yan (2013)	48	47	50	45	41.5 ± 3.1	42.7 ± 4.2	12	Dan-ning tablet + CDs	CDs	Clinical effective rate, ALT, TC, TG, TBIL
15	Zhang xiyun (2020)	48	48	39	57	44.15 ± 7.52	43.25 ± 7.09	12	Dan-ning tablet + CDs	CDs	Clinical effective rate, ALT, AST, *γ*-GT, TC, TG
16	Wang zhiling (2014)	127	116	160	83	46.5 ± 7.5	47 ± 7.4	12	Dan-ning tablet + CDs	CDs	Clinical effective rate, ALT, AST, TC, TG
17	Li bing (2018)	52	52	45	59	41.82 ± 8.63	40.45 ± 8.35	12	Dan-ning tablet + CDs	CDs	Clinical effective rate, ALT, AST, *γ*-GT, TC, TG, LDL, HDL, TBIL
18	Fan qiaowen (2019)	50	50	72	28	55.5 ± 1.8	56 ± 1.8	12	Dan-ning tablet + CDs	CDs	Clinical effective rate, ALT, *γ*-GT, TC, TG
19	Ji guang (2008)	107	33	102	38	48.37 ± 9 .60	44.43 ± 10.40	12	Dan-ning tablet + CDs	CDs	Clinical effective rate, ALT, AST, *γ*-GT, TC, TG
20	Song shoulong (2018)	45	45	53	37	42.35 ± 4.26	42.31 ± 4.21	6	Dang-fei-Li-Gan-Ningcapsule + CDs	CDs	Clinical effective rate, ALT, AST, TBIL
21	Li chaomin (2012)	113	114	150	77	45.5 ± 11.8	46.7 ± 10.8	12	Dang-fei-Li-Gan-Ningcapsule + CDs	CDs	Clinical effective rate, ALT, AST, TC, TG, LDL, HDL
22	LI guozheng (2009)	40	40	—		—		12	Dang-fei-Li-Gan-Ningcapsule + CDs	CDs	Clinical effective rate, ALT, AST, TC, TG, LDL, HDL
23	Zhang xue (2015)	30	30	29	31	20∼55	18∼60	24	Dang-fei-Li-Gan-Ningcapsule + CDs	CDs	Clinical effective rate, ALT, TC, TG
24	Li li (2010)	45	45	54	36	18∼56	26∼61	24	Qiang-Gancapsule + CDs	CDs	Clinical effective rate, ALT, AST, TC, TG, *γ*-GT
25	Tang liwei (2019)	58	58	—		—		24	Qiang-Gancapsule + CDs	CDs	Clinical effective rate, ALT, AST, TC, TG, *γ*-GT
26	Yao zhongcai (2011)	75	75	88	62	46.7 ± 11.8	45.3 ± 12.6	12	Qiang-Gancapsule + CDs	CDs	Clinical effective rate, ALT, AST, TC, TG, *γ*-GT
27	Bai lihua (2016)	45	45	55	35	23～67	21～64	24	Qiang-Gancapsule + CDs	CDs	Clinical effective rate, ALT, AST, *γ*-GT
28	Wang xiuqin (2019)	119	119	89	149	45.62 ± 10.21	44.53 ± 8.87	12	Qiang-Gancapsule + CDs	CDs	Clinical effective rate, ALT, AST, *γ*-GT
29	Liu hongfen (2016)	32	30	34	28	39.5 ± 10.2	39.1 ± 9.1	12	Qiang-Gancapsule + CDs	CDs	Clinical effective rate, ALT, *γ*-GT, TC
30	Chen zexiong (2006)	64	58	77	45	42.5	45.8	12	Qiang-Gancapsule + CDs	CDs	Clinical effective rate, ALT, AST, TC, TG, *γ*-GT
31	Wang yanping (2015)	150	150	128	172	35.8 ± 3.7	37.2 ± 3.3	24	Qiang-Gancapsule + CDs	CDs	Clinical effective rate, ALT, AST, TC, TG, *γ*-GT
32	Han qing (2019)	90	90	114	66	43.64 ± 5.82	41.28 ± 5.35	8	Hua-zhi-rou-Gangranule + CDs	CDs	Clinical effective rate, ALT, AST, TC, TG, LDL, HDL
33	Li haixia (2017)	57	58	62	53	41.3 ± 4.8	42.3 ± 5.4	12	Hua-zhi-rou-Gangranule + CDs	CDs	Clinical effective rate, ALT, AST, TC, TG, *γ*-GT
34	Zhang chunming (2019)	30	30	37	23	52.0 ± 10.8	52.3 ± 10.4	—	Hua-zhi-rou-Gangranule + CDs	CDs	Clinical effective rate
35	Wang xiling (2018)	57	57	74	40	48.5 ± 8.1	49.4 ± 6.1	12	Hua-zhi-rou-Gangranule + CDs	CDs	Clinical effective rate, ALT, AST, TC, TG
36	Guo suicheng (2013)	60	60	72	48	37 ± 4.21		8	Hua-zhi-rou-Gangranule + CDs	CDs	Clinical effective rate, ALT, AST, *γ*-GT
37	Luo qing (2019)	50	50	58	42	36.76 ± 1.58	36.54 ± 1.37	8	Hua-zhi-rou-Gangranule + CDs	CDs	Clinical effective rate, ALT, AST, *γ*-GT, TC, TG, LDL, HDL, TBIL
38	Fang junwei (2014)	132	131	178	85	42.84 ± 7.49	41.90 ± 8.32	12	Hua-zhi-rou-Gangranule + CDs	CDs	Clinical effective rate, ALT, AST, TC, TG, LDL, HDL
39	Lin yudong (2013)	60	60	90	30	43.3 ± 5.8	42.8 ± 6.3	12	Hua-zhi-rou-Gangranule + CDs	CDs	Clinical effective rate, ALT, AST, TC, TG
40	Yu yang (2014)	30	30	34	26	44.7 ± 9.3	43.7 ± 9.2	12	Hua-zhi-rou-Gangranule + CDs	CDs	Clinical effective rate, ALT, AST, TC, TG, *γ*-GT
41	Yang shushan (2015)	90	90	118	62	49.5 ± 7.5	50.4 ± 7.1	12	Hua-zhi-rou-Gangranule + CDs	CDs	Clinical effective rate, ALT, AST, TC, TG
42	Xu junlin (2018)	70	70	80	60	44.7 ± 7.5	43.5 ± 7.1	12	Hua-zhi-rou-Gangranule + CDs	CDs	Clinical effective rate, ALT, AST, TC, TG
43	Nan (2020)	40	40	31	49	37.2 ± 9.4		8	Hua-zhi-rou-Gangranule + CDs	CDs	Clinical effective rate, ALT, AST, TC, TG, *γ*-GT

*Note.* CDs: Chemical drugs, ALT: Alanine aminotransferase, AST: Aspartate aminotransferase, TC: Total cholesterol, TG: Triglycerides, *γ*-GT: *γ*-glutamyltranspeptidase, LDL: Low-density lipoprotein, HDL: High-density lipoprotein, TBIL: Total bilirubin.

**Table 2:** Results of the network meta-analysis of the effective rate.

CDs					
**0.26 (0.10, 0.67)**	DHLD + CDs				
**0.19 (0.12, 0.31)**	0.76 (0.26, 2.21)	DN + CDs			
**0.21 (0.09, 0.46)**	0.81 (0.23, 2.83)	1.07 (0.42, 2.71)	DFLGN + CDs		
**0.44 (0.27, 0.74)**	1.74 (0.58, 5.17)	**2.30 (1.15, 4.59)**	2.15 (0.84, 5.51)	QG + CDs	
**0.27 (0.17, 0.43)**	1.06 (0.36, 3.09)	1.40 (0.73, 2.71)	1.31 (0.52, 3.29)	0.61 (0.31,1.21)	HZRG + CDs

*Note.* Significant effects are printed in bold.

**Table 3:** SUCRA for outcomes.

	Clinical effective rate (%)	ALT (%)	AST (%)	TC (%)	TG (%)
^DHLD + CDs^	^61.1^	^55.4^	^77.5^	^55.8^	^49.9^
^DN + CDs^	^81.8^	^85.5^	^47.1^	^42.6^	^60.6^
^DFLGN + CDs^	^74.9^	^38.8^	^83.6^	^76.3^	^40.6^
^QG + CDs^	^25.9^	^62.3^	^10.0^	^37.4^	^68.4^
^HZRG + CDs^	^56.2^	^55.9^	^70.4^	^87.1^	^79.9^
^CDs^	^0.1^	^2.0^	^11.4^	^1.0^	^0.6^

**Table 4:** Results of the network meta-analysis of the ALT.

CDs					
11.05 (−0.37, 22.48)	DHLD + CDs				
**15.81 (10.05, 21.57)**	4.76 (−7.97, 17.48)	DN + CDs			
8.00 (−2.68, 18.67)	−3.06 (−18.64, 12.53)	−7.81 (−19.94, 4.32)	DFLGN + CDs		
**12.20 (4.42, 19.99)**	1.15 (−12.61, 14.90)	−3.61 (−13.29, 6.07)	4.21 (−9.01, 17.42)	QG + CDs	
**11.23 (4.85, 17.62)**	0.18 (−12.85, 13.20)	−4.58 (−13.18, 4.02)	3.23 (−9.20, 15.67)	−0.97 (−11.04, 9.10)	HZRG + CDs

*Note.* Significant effects are printed in bold.

**Table 5:** Results of the network meta-analysis of the AST.

CDs					
13.45 (3.61,23.28)	DHLD + CDs				
**7.43 (1.95, 12.91)**	−6.02 (−17.24, 5.21)	**DN** **+** **CDs**			
**14.94 (4.77, 25.11)**	1.50 (−12.62, 15.62)	7.51 (−4.04, 19.07)	**DFLGN** **+** **CDs**		
−0.62 (−7.48,6.25)	−**14.06 (**−**26.02,** −**2.10)**	−8.05 (−16.83, 0.74)	−15.56 (−27.83, −3.29)	**QG** **+** **CDs**	
**11.63 (6.25, 17.02)**	−1.81 (−12.99, 9.36)	4.20 (−3.48, 11.89)	−3.31 (−14.81, 8.20)	**12.25 (3.53, 20.98)**	**HZRG** **+** **CDs**

*Note.* Significant effects are printed in bold.

**Table 6:** Results of the network meta-analysis of the TC.

CDs					
0.63 (−0.03, 1.29)	**DHLD** **+** **CDs**				
**0.50 (0.18, 0.82)**	−0.13 (−0.86, 0.60)	**DN** **+** **CDs**			
**0.87 (0.28, 1.45)**	0.24 (−0.65, 1.12)	0.36 (−0.31, 1.03)	**DFLGN** **+** **CDs**		
**0.45 (0.04, 0.87)**	−0.18 (−0.96, 0.60)	−0.05 (−0.58, 0.48)	−0.41 (−1.13, 0.31)	**QG** **+** **CDs**	
**0.97 (0.56, 1.39)**	0.34 (−0.44, 1.12)	0.47 (−0.05, 1.00)	0.11 (−0.61, 0.83)	0.52 (−0.07, 1.11)	**HZRG** **+** **CDs**

*Note.* Significant effects are printed in bold.

**Table 7:** Results of the network meta-analysis of the TG.

CDs					
0.42 (0.04, 0.80)	DHLD + CDs				
**0.49 (0.30, 0.68)**	0.07 (−0.36, 0.49)	DN + CDs			
**0.36 (0.03, 0.70)**	−0.06 (−0.56, 0.45)	−0.12 (−0.51, 0.26)	DFLGN + CDs		
**0.53 (0.26, 0.79)**	0.11 (−0.36, 0.57)	0.04 (−0.29, 0.37)	0.16 (−0.26, 0.59)	QG + CDs	
**0.59 (0.35, 0.83)**	0.17 (−0.28, 0.62)	0.10 (−0.21, 0.41)	0.22 (−0.19, 0.64)	0.06 (−0.30, 0.42)	**HZRG** **+** **CDs**

*Note.* Significant effects are printed in bold.

## Data Availability

The data used to support the findings of this study are available from the corresponding author upon request.

## Abbreviations

CDs: Chemical drugs
NAFLD: Nonalcoholic fatty liver disease
CPMs: Chinese patent medicines
PRCTs: Pragmatic randomized controlled trials
DHLD: Da-huang-Li-dan capsule
DN: Dan-Ning tablet
DFLGN: Dang-fei-li-gan-ning capsule
QG: Qiang-gan capsule
HZRG: Hua-zhi-rou-gan granule
TCM: Traditional Chinese medicine.
